The article "Risk Factor Analysis for Predicting the Onset of Rotator Cuff Calcific Tendinitis Based on Artificial Intelligence" was retracted in 2023. Reasons: signs of a paper mill; compromised peer review; unreliable results or conclusions.

# Risk Factor Analysis for Predicting the Onset of Rotator Cuff Calcific Tendinitis Based on Artificial Intelligence

**DOI:** 10.1155/2022/8978878

**Published:** 2022-04-11

**Authors:** Shengtao Dong, Jie Li, Haozong Zhao, Yuanyuan Zheng, Yaoning Chen, Junxi Shen, Hua Yang, Jieyang Zhu

**Affiliations:** ^1^Department of Spine Surgery, The Second Affiliated Hospital of Dalian Medical University, Dalian 116023, China; ^2^Department of Gastrointestinal Surgery, The Second Affiliated Hospital of Dalian Medical University, Dalian 116023, China; ^3^Department of Oncology, The Second Affiliated Hospital of Dalian Medical University, Dalian 116023, China; ^4^Department of Otolaryngology, Head and Neck Surgery, Second Affiliated Hospital of Dalian Medical University, Dalian 116000, China

## Abstract

**Background:**

Symptomatic rotator cuff calcific tendinitis (RCCT) is a common shoulder disorder, and approaches combined with artificial intelligence greatly facilitate the development of clinical practice. Current scarce knowledge of the onset suggests that clinicians may need to explore this disease thoroughly.

**Methods:**

Clinical data were retrospectively collected from subjects diagnosed with RCCT at our institution within the period 2008 to 2020. A standardized questionnaire related to shoulder symptoms was completed in all cases, and standardized radiographs of both shoulders were extracted using a human-computer interactive electronic medical system (EMS) to clarify the clinical diagnosis of symptomatic RCCT. Based on the exclusion of asymptomatic subjects, risk factors in the baseline characteristics significantly associated with the onset of symptomatic RCCT were assessed via stepwise logistic regression analysis.

**Results:**

Of the 1,967 consecutive subjects referred to our academic institution for shoulder discomfort, 237 were diagnosed with symptomatic RCCT (12.05%). The proportion of women and the prevalence of clinical comorbidities were significantly higher in the RCCT cohort than those in the non-RCCT cohort. Stepwise logistic regression analysis confirmed that female gender, hyperlipidemia, diabetes mellitus, and hypothyroidism were independent risk factors for the entire cohort. Stratified by gender, the study found a partial overlap of risk factors contributing to morbidity in men and women. Diagnosis of hyperlipidemia, diabetes mellitus, and hypothyroidism in male cases and diabetes mellitus in female cases were significantly associated with symptomatic RCCT.

**Conclusion:**

Independent predictors of symptomatic RCCT are female, hyperlipidemia, diabetes mellitus, and hypothyroidism. Men diagnosed with hyperlipidemia, diabetes mellitus, and hypothyroidism are at high risk for symptomatic RCCT, while more medical attention is required for women with diabetes mellitus. Artificial intelligence offers pioneering innovations in the diagnosis and treatment of musculoskeletal disorders, and careful assessment through individualized risk stratification can help predict onset and targeted early stage treatment.

## 1. Introduction

Rotator cuff calcific tendinitis (RCCT) is a disease associated with pain and limitation of motion due to calcium deposits in the tendon [1]. Previous literature suggests that approximately 2.7%–36% of the global population is afflicted by RCCT, with 30–60 years women being the vulnerable population for the disease [2–7]. The supraspinatus tendon is the most frequent target of the lesion, followed by the infraspinatus and subscapularis tendons [8].

There are various clinical symptoms of RCCT due to pathological changes. RCCT can be divided into four stages according to the pathological stage: precalcification, calcification, resorption, and repair. Precalcification is mainly manifested by the appearance of fibrocartilage in the tendon, and patients usually have no corresponding clinical symptoms at this time. Calcification phase is the stage of calcium salt deposition in the tendon. During the resorption phase of calcification, the patient experiences severe pain and limitation of motion for several weeks due to increased pressure in the tendon sheath due to subacromial capsular edema and extravasation of calcium salt crystals. The repair phase reflects the self-healing nature of RCCT, with tendon healing, disappearance of the calcified foci, and rearrangement of the collagen fibers, resulting in a significant reduction or even disappearance of symptoms compared with the previous phase [9, 10]. Given the dynamic clinical picture of RCCT, definitive radiological findings are a necessary component of the diagnosis, including standard X-rays and susceptibility-weighted imaging (SWI) MRI [11]. Previous literature has shown the use of artificial intelligence to analyze the clinical characteristics of patients with common disorders and thus found positive correlations between onset and prognosis [12–14].

Although published studies have highlighted a wide range of risk factors for the onset of calcific rotator cuff tendinitis [15–17], including endocrine disorders [18], hyperlipidemia [4], and sports strain [19], the etiology of symptomatic RCCT is currently inconclusive. A study by Witte et al. published in 2016 reported risk factors associated with outcomes, female gender, dominant arm involvement, bilateral disease, longer duration of symptoms, and multiple calcifications were associated with poorer outcomes. In this work, we report the incidence of RCCT based on human-computer interaction data extraction by selecting target cases from our institution's electronic medical system and analysis risk factors significantly associated with asymptomatic RCCT from routine clinical data.

## 2. Materials and Methods

### 2.1. Patient Population

Between January 2008 and December 2020, all patients referred to our academic institution for shoulder discomfort were routinely screened for evaluation for inclusion in the study. Inclusion criteria were as follows: (1) radiological evidence of shoulder pain and limited motion; (2) age between 18 and 60 years at diagnosis; and (3) available clinical information. Exclusion criteria were as follows: (1) prior shoulder trauma or shoulder surgery; (2) diagnosis of malignancy; and (3) unavailable X-ray results.

Clinical characteristics and radiological reports were reviewed and recorded through an electronic medical system (EMS) [20], including age at diagnosis, sex, BMI at diagnosis, smoking status, alcohol use status, physical demand (light/heavy), diabetes mellitus, hypertension, cardiovascular disease, hyperlipidemia, and hypothyroidism. The diagnostic criteria for hyperlipidemia were the presence of the diagnosis in the medical record or meeting one or more of the following criteria from the American Association of Clinical Endocrinologists' Guidelines for the Management of Dyslipidemia and Prevention of Atherosclerosis: total cholesterol (TC) ≥6.22 mmol/dL; high-density lipoprotein cholesterol (HDL-C) <1.04 mmol/dL; low-density lipoprotein cholesterol (LDL- C) ≥4.14 mmol/dL; and triglycerides (TG) ≥2.26 mmol/dL.

Radiological diagnosis was evaluated independently and blinded by two experienced investigators (Figure 1). In case of disagreement, shoulder MRI was added and the radiological results were re-evaluated in a comprehensive approach by a senior musculoskeletal radiologist. To clarify the condition of calcification around symptomatic RCCT, its radiological diagnosis was defined as any calcification in anteroposterior (internal and external rotation) and axial views including the subscapularis, the infraspinatus, and teres minor tendons.

### 2.2. Statistical Analysis

Pearson chi-square test was used to test continuous data (*n* ≥ 40), with continuity correction if 1 ≤ *T* < 5 and Fisher's exact test if *T* < 1. Independent sample *t*-test was performed for normally distributed categorical data; otherwise, Mann–Whitney *U* test was performed. Stepwise logistic regression analysis was used to determine independent risk factors for the onset of RCCT. All statistics were performed using SPSS version 22.0 (IBM SPSS, Armonk, New York). The abovementioned analysis results were considered statistically significant only in cases of *P* < 0.05.

## 3. Results

There were 1967 patients enrolled for shoulder discomfort, of which 237 were diagnosed with symptomatic RCCT and 1730 were classified as other shoulder disorders. In terms of clinical comorbidities, 87 patients were diagnosed with hyperlipidemia (22 in the RCCT cohort and 65 in the control cohort), 294 with hypertension (33 in the RCCT cohort and 261 in the control cohort), 253 with diabetes mellitus (48 in the RCCT cohort and 205 in the control cohort), 144 with hypothyroidism (29 in the RCCT cohort and 115 in the control 115 in the cohort), and 102 with cardiovascular disease (8 in the RCCT cohort and 94 in the control cohort). Women proved to be the more common group, with 172 of 1396 female patients enrolled (72.57%) diagnosed with RCCT and 65 of 571 male patients (27.43%) with RCCT. Compared with the control group, the RCCT cohort had a higher prevalence of clinical comorbidities (hyperlipidemia, diabetes mellitus, and hypothyroidism). This finding suggests a mechanism of interaction between RCCT and other comorbidities. However, this study did not find statistically significant age at diagnosis, BMI, smoking status, alcohol consumption status, hypertension, cardiovascular disease, and exercise requirements (Table 1).

Stepwise logistic regression analysis was used to examine the independent risk factors significantly associated with the development of symptomatic RCCT. Univariate logistic regression initially screened for variables that were statistically different in the overall cohort, including female, smoking status, hyperlipidemia, hypertension, diabetes mellitus, and hypothyroidism. Multivariate analysis review confirmed that female gender, hyperlipidemia, diabetes mellitus, and hypothyroidism still demonstrated statistically significant differences (Table 2). Our finding that gender plays an extremely important role in predicting symptomatic RCCT was corroborated by the previous literature. After risk stratification of the overall cohort according to gender, the statistical predictors for the male cohort were hyperlipidemia, diabetes mellitus, and hypothyroidism (Table 3). In comparison to the overall cohort and statistical indicators of patient morbidity in men, only the occurrence of diabetes showed a significant effect on morbidity in females after applying the same analysis to their cases (Table 4).

## 4. Discussion

Since Uhthoff first reported the pathological cycle of calcific tendinitis in 1997, this disease caused by calcium phosphate crystalline calcium salt deposits has become increasingly recognized [21]. Because the onset of calcific tendinitis occurs through several different pathologic scenarios, patients often complain in a variety of ways, including painless asymptomatic and mildly painful phases, as well as intense painful, limited movement phases. Given the lack of adequate clinical cues, patients in the asymptomatic phase are usually not referred to a medical center until pain develops. In symptomatic RCCT, definitive radiological findings combined with clinical complaints can lead to a definitive diagnosis [14, 22, 23]. In this first study involving a large cohort of RCCT patients, we found an association between morbidity and common clinical routine parameters that may help achieve secondary prevention of RCCT.

The female gender, especially those aged 30–60 years, is a more susceptible cohort for RCCT compared with the male gender. As found in previous reports, RCCT occurs more frequently in women, accounting for approximately 52%–79% of the total incidence [24–26]. Our study is consistent with published findings that a 72.57% prevalence rate confirms that women suffer from more pain. To further clarify the potential association between gender and the onset of symptomatic RCCT, Harvie and colleagues introduced an acceptable explanation for the effect of sex hormones on the function of the tendons around the shoulder joint [18]. On the one hand, the joints are more lax in women compared to men, and on the other hand, sex hormone-induced neurogenic inflammation leads to stiffer tendons in women [18]. However, it is slightly reluctant to infer a direct correlation between females and unfavorable clinical symptoms with the current evidence. In this regard, we consider that calcification diameter may be another relevant factor associated with shoulder pain, and previous findings in the literature confirm that symptoms are more often seen in calcification deposits larger than 1 cm [25]. Therefore, estrogen in women may accelerate the deposition of calcium salts compared with asymptomatic or male patients, shortening the time for calcification to reach the pain threshold size. In addition to this, in a 14-year-long follow-up by Witte et al., female gender was significantly associated with inferior clinical long-term outcomes [25]. Therefore, it is reasonable to suppose that the onset of RCCT is not only gender-selective but also that the self-limiting nature of this disease is not adequately characterized compared with its counterpart, and that the prognosis of female patients did not show the expected improvement at decade follow-up [27]. To distinguish the key role played by gender, we stratified this risk, with people of different genders showing various responses to risk factors. Men diagnosed with hyperlipidemia, diabetes, and hypothyroidism are at high risk for symptomatic RCCT, while women with diabetes are more likely to develop symptomatic RCCT.

As a common co-existing metabolic disorder, adults with a diagnosis of diabetes bear a greater risk of skeletal muscle disease [28]. In general, it is well established that disruption of shoulder tendon homeostasis can be observed in diabetic tendinopathy, manifested by shoulder pain, joint stiffness, limitation of motion, rotator cuff tears, and tendon calcification. The underlying molecular mechanisms of these pathological deteriorations can be attributed to abnormalities in collagen fibers, including alterations in number, morphology, and disorganization [29]. A national population study by Su et al. confirmed that the risk of secondary calcific tendonitis in patients diagnosed with either type 1 or type 2 diabetes was about 27%. Their hypothesis for this was that diabetes-induced vascular compromise and hyperglycemic exposure; the former may reduce the supply of nutrients and oxygen to connective tissue, thus causing degeneration and promoting calcification deposits, and the latter may lead to glycosylation of extracellular proteins, thus altering the biomechanical environment and possibly promoting calcification of connective tissue [30]. Furthermore, distinguishing between symptomatic and asymptomatic RCCT, after searching the literature, we found that Siu et al. reported elevated subacromial fluid IL-1*β* levels in diabetic patients with shoulder pain and shoulder stiffness, which may be strong evidence to support the diagnosis of symptomatic RCCT [31].

Hyperlipidemia, a systemic metabolic disorder, has adverse effects on the cardiovascular and musculoskeletal systems. The mechanical properties of tendons are reduced by excessive accumulation of lipids in the extracellular matrix, and fatty infiltration can impair post-surgical tendon-bone healing and clinical outcomes [3]. A significantly higher incidence of calcific tendinitis was reported after 11 years of follow-up in patients with hyperlipidemia by Lin et al. Meanwhile, treatment of hyperlipidemia served as an effective protective factor against RCCT [32]. Substantial research evidence suggests that statins can decrease lipid levels while simultaneously demonstrating the anti-inflammatory qualities associated with hyperlipidemia, facilitating the treatment and control of inflammatory musculoskeletal disorders, such as RCCT [33].

Thyroxine is well known to be central to both collagen synthesis and matrix metabolism. Hypothyroidism leads to accumulation of glycosaminoglycans in the extracellular matrix and exacerbates tendon calcification. In patients with RCCT in combination with hypothyroidism, treatment of the primary hypothyroidism can provide significant relief of secondary shoulder pain [18, 34]. A clinical study has demonstrated that patients diagnosed with RCCT suffer more from co-existing hypothyroidism. Calcified tendons in hypothyroidism generally continue to impair shoulder function for up to 5 years compared with nonhypothyroid patients who recover on their own within 1 year [18].

The current study has some limitations. This single-center retrospective study which only reflects the case characteristics of this region may be subject to selection bias. Although we have tried to screen for routine clinical indicators as much as possible, other causes of symptomatic RCCT onset may still be missed. Meanwhile, as patient information is collected from EMS, potential target cases may be excluded due to poorly written diagnoses. Finally, the selected patients were all hospitalized, so this study sample is not representative of the characteristics of mild disease overall. The selection of controls in the medical record system did not allow for the identification of absolutely “healthy” blank controls, and the use of other shoulder diseases as controls may have artificially influenced the distribution of the number and degree of certain factors in the control group, such as age distribution, and thus prevented accurate investigation of these factors in this study.

## 5. Conclusion

The results from our clinical study indicated that female gender, diabetes mellitus, hyperlipidemia, and hypothyroidism were significant risk factors for the unfavorable clinical symptoms in patients with RCCT. Our work serves as a reference for aggressive prevention and standardized treatment of RCCT, and clinicians can thoroughly investigate and understand the pathogenesis of this disease.

## Figures and Tables

**Figure 1:** Anteroposterior X-rays of a 45-year-old female patient with shoulder pain for 5 months due to RCCT.

**Table 1:** Comparison of the baseline clinical characteristics.

	All subjects	RCCT cohort	Control cohort	*p*
Number of patients	1967	237	1730	
Age at diagnosis (years)	45.2	43.6	45.7	0.432
Sex (%)				0.038
Female	1396 (70.97)	172 (72.57)	1224 (70.75)	
Male	571 (29.03)	65 (27.43)	506 (29.25)	
BMI (kg/m^2^)	21.32 ± 1.84	20.44 ± 1.71	21.44 ± 2.34	0.173
Smoking status (%)	355 (18.05)	50 (21.10)	305 (17.63)	0.346
Alcohol use status (%)	318 (16.17)	41 (17.30)	277 (16.01)	0.257
Hyperlipidemia (%)	87 (4.42)	22 (9.28)	65 (3.76)	0.022
Hypertension (%)	294 (14.95)	33 (13.92)	261 (15.09)	0.075
Diabetes mellitus (%)	253 (12.86)	48 (20.25)	205 (11.85)	<0.001
Hypothyroidism (%)	144 (7.32)	29 (12.24)	115 (6.65)	0.009
Cardiovascular disease (%)	102 (5.19)	8 (3.38)	94 (5.43)	0.731
Physical demand (%)				0.517
Light	1088 (55.31)	131 (55.27)	957 (55.32)	
Hard	879 (44.69)	106 (44.73)	773 (44.68)	

Data are reported as mean (±SD) or frequency/ratio. BMI: body mass index; SD: standard deviation.

**Table 2:** Relationship between variables and RCCT by stepwise logistic regression analysis.

	Univariable			Multivariable		
	OR	95% CI	*p*	OR	95% CI	*p*
*Sex*						
Male	Ref	Ref	Ref	Ref	Ref	Ref
Female	3.909	3.581–5.617	<0.001	2.654	1.189–3.912	0.011
Smoking status	1.073	1.009–1.104	0.044	1.958	1.174–2.911	0.265
Hyperlipidemia	1.124	1.031–1.226	0.004	1.089	1.019–1.466	0.010
Hypertension	2.364	1.057–3.125	0.039	1.307	1.076–1.891	0.157
Diabetes mellitus	1.718	1.035–4.509	<0.001	3.166	1.922–5.011	0.002
Hypothyroidism	1.708	1.378–2.141	0.015	1.478	1.091–1.974	0.025

OR: odds ratio; 95% CI: 95% confidence interval.

**Table 3:** Multivariate logistic analysis results among male patients.

	Univariable			Multivariable		
	OR	95% CI	*p*	OR	95%CI	*p*
Hyperlipidemia	1.802	1.646–2.561	0.007	2.171	1.157–2.879	0.029
Diabetes mellitus	1.372	1.107–3.509	<0.001	2.025	1.203–3.952	0.009
Hypothyroidism	1.802	1.158–2.087	0.008	3.600	1.118–8.063	0.036

**Table 4:** Multivariate logistic analysis results among female patients.

	Univariable			Multivariable		
	OR	95% CI	*p*	OR	95%CI	*p*
Hyperlipidemia	2.071	0.714–3.009	0.014	2.595	0.890–2.527	0.180
Diabetes mellitus	1.614	1.302–5.625	<0.001	3.422	1.227–8.785	0.006
Hypothyroidism	1.113	1.021–2.069	0.031	2.101	1.007–3.005	0.220

## Data Availability

The data used to support the findings of this study are available from the corresponding author upon request.

## Abbreviations

RCCT: Rotator cuff calcific tendinitis
AP: Anteroposterior
SWI: Susceptibility-weighted imaging
MRI: Magnetic resonance imaging
BMI: Body mass index
TC: Total cholesterol
HDL-C: High-density lipoprotein cholesterol
LDL-C: Low-density lipoprotein cholesterol
TG: Triglycerides
SD: Standard deviation
EMS: Electronic medical system
AP: Anteroposterior
OR: Odds ratio
95% CI: 95% confidence interval.
